The article "An Analytical Study of Speech Pathology Detection Based on MFCC and Deep Neural Networks" was retracted in 2023. Reasons: signs of a paper mill; compromised peer review; unreliable results or conclusions.

# An Analytical Study of Speech Pathology Detection Based on MFCC and Deep Neural Networks

**DOI:** 10.1155/2022/7814952

**Published:** 2022-04-04

**Authors:** Mohammed Zakariah, Reshma B, Yousef Ajmi Alotaibi, Yanhui Guo, Kiet Tran-Trung, Mohammad Mamun Elahi

**Affiliations:** ^1^Department of Computer Science, College of Computer and Information Sciences, King Saud University, P.O. Box 57168, Riyadh 21574, Saudi Arabia; ^2^Division of Electronics Engineering, School of Engineering, Cochin University of Science and Technology, India; ^3^Department of Computer Engineering, College of Computer and Information Sciences, King Saud University, P.O. Box 57168, Riyadh 21574, Saudi Arabia; ^4^University of Illinois Springfield, USA; ^5^Faculty of Computer Science, Ho Chi Minh City Open University, 97 Vo Van Tan, Ward Vo Thi Sau, District 3, Ho Chi Minh City Code postal: 70000, Vietnam; ^6^Department of Computer Science and Engineering, United International University, Dhaka, Bangladesh

## Abstract

Diseases of internal organs other than the vocal folds can also affect a person's voice. As a result, voice problems are on the rise, even though they are frequently overlooked. According to a recent study, voice pathology detection systems can successfully help the assessment of voice abnormalities and enable the early diagnosis of voice pathology. For instance, in the early identification and diagnosis of voice problems, the automatic system for distinguishing healthy and diseased voices has gotten much attention. As a result, artificial intelligence-assisted voice analysis brings up new possibilities in healthcare. The work was aimed at assessing the utility of several automatic speech signal analysis methods for diagnosing voice disorders and suggesting a strategy for classifying healthy and diseased voices. The proposed framework integrates the efficacy of three voice characteristics: chroma, mel spectrogram, and mel frequency cepstral coefficient (MFCC). We also designed a deep neural network (DNN) capable of learning from the retrieved data and producing a highly accurate voice-based disease prediction model. The study describes a series of studies using the Saarbruecken Voice Database (SVD) to detect abnormal voices. The model was developed and tested using the vowels /a/, /i/, and /u/ pronounced in high, low, and average pitches. We also maintained the “continuous sentence” audio files collected from SVD to select how well the developed model generalizes to completely new data. The highest accuracy achieved was 77.49%, superior to prior attempts in the same domain. Additionally, the model attains an accuracy of 88.01% by integrating speaker gender information. The designed model trained on selected diseases can also obtain a maximum accuracy of 96.77% (cordectomy × healthy). As a result, the suggested framework is the best fit for the healthcare industry.

## 1. Introduction

In several occupations that need impeccable pronunciation, voice and speech are vital. It is also the most convenient method of interpersonal interaction. Language difficulties can result in incomprehensible conversation and misunderstandings. Tissue disease, systemic alterations, mechanical stress, surface frustration, tissue modifications, neurological and muscle abnormalities, and other variables like air pollution, smoking, and stress can all induce vocal disease [1, 2]. The vocal cords' movement, functioning, and morphology are compromised by voice pathology, resulting in uneven pulsations and improved auditory noise. This type of speech sounds stressed, tough, feeble, and panting [3], which adds significantly to the overall bad vocal quality [4, 5].

Currently, existing voice pathology diagnosis tools are based on personal factors. Auditory-perceptual assessment in hospitals, extensively used for pictorial laryngostroboscopy evaluation, is a form of subjective assessment [6]. In addition, different clinical assessments are used to grade the rate of severity diagnosis for auditory-perceptual characteristics [7]. Nevertheless, such assessment approaches are factor-sensitive, time-consuming, and difficult [8]. Furthermore, such procedures necessitate a physical evaluation of the patient in the clinic, which may be problematic for serious illnesses.

Consuming a computer-aided device to recognize and evaluate speech sounds without surgical interference is a form of objective assessment. The phoniatric condition for appropriate and pathological vocal production corresponds well with the acoustic properties, which offers a physical explanation of the waveforms created and transmitted by the vocal organs. Additionally, audio signal processing stimulates the development of more recognizable human vocal characteristics. It enables an accurate, objective evaluation of voice and speech disorders, even in the presence of audible noises [9]. These evaluation approaches are not subjective because they do not rely on human opinion. They are also simple because the voice recordings may be viewed remotely using different Internet recording applications. Consequently, some study findings, such as [10], have created a voice computation approach to calculate voice pathology elements that can be effectively combined with a machine learning method for automatically detecting voice pathology in one structure to precisely differentiate healthy people from individuals with audio pathologies.

Typically, conventional and clinically interpretable [5] acoustic characteristics were calculated preliminary to pathology identification [11, 12]. Following extracting features, several traditional algorithms were applied to determine the existence of vocal pathology. Extreme learning machine (ELM) [13], support vector machine (SVM) [14], and Gaussian mixture model (GMM) are among the machine learning methods that have been used in voice recognition of vocal pathology structures [15]. Hence, machine learning procedures have demonstrated their efficacy and proficiency in distinguishing diseased sounds from regular speech. Conventional and clinically interpretable [5] acoustic characteristics were calculated preliminary to pathology identification [12]. The limitations of voice pathology detection systems can be summarized as follows: Most studies focused only on a single dialogue task, primarily the continuous phonation of the vowel /a/ which examined only one aspect of speech. Most studies examined datasets from one to three databases that were confined to a subset of vocal disorders (MEEI, SVD, and AVPD). As a result, there are just a few voice databases for healthy and sick samples. The bulk of the research concentrates solely on the exposure of speech pathology while ignoring pathological categorization jobs. Voice disorder structures are assessed exclusively by precision, specificity, and sensitivity.

As a result, it is critical to create a dependable vocal pathology recognition structure based on machine learning to handle these challenges. In this study, we attempted to investigate the performance of the deep neural network (DNN) on the mel spectrogram and several other features. This study makes the following contributions:

- We created a deep neural network (DNN) to identify and classify pathological and healthy voices
- The suggested approach employs SVD healthy and pathological voice samples, taking into account phrases and vowels /a/, /i/, and /u/ generated in three distinct pitches
- The suggested method trains and evaluates the DNN by utilizing a large number of healthy and pathological speech samples compared to previous works in the domain
- The present study attempted to illustrate the impact of gender knowledge on correctly identifying pathological and healthy classes
- The algorithm also attempts to comprehend how the model generalizes to the “continuous sentence” samples
- The research also attempted to do a multiclass classification into two pathological classes and one healthy class to determine if the information and model were competent enough for the operation

The remainder of the paper is laid out as follows. The previous literature relevant to this work is presented in Section 2. The complete methodology is described in Section 3, which includes the dataset used in this work and other operations like extraction of features, proposed network architecture, and the training pipeline. The results are presented in Section 4, followed by a discussion in Section 5. Conclusions are drawn in Section 6, followed by references.

## 2. Literature Review

The study on automated speech pathology identification concentrated on identifying new variables that may distinguish between normal and abnormal voices or even assess their quality, as well as alternative methodologies for categorization.

Many auditory elements have been studied in the literature, each with a distinct concentration, to discover the specific qualities of the sound. Many approaches based on signal statistics have already been presented in the literature, notably cycle-to-cycle fluctuations in the time sphere [16]. Calculations constructed on fundamental frequency, assessment of the period-to-period variation of the tone interval (jitter coefficient), and demographics are the key aspects of research and pathological speech assessment. Regularity disruption and amplitude inflection (shimmer coefficients) have been employed in the study and assessment of speech quality, like shimmer, jitter, harmonic noise ratio, signal-to-noise ratio, and glottal-to-noise ratio [17–20]. The excitation of the signal is often considered in the identification of vocal fold disease [21]. Commercial voice recognition tools have made tools for voice-based disruption broadly available. The fundamental frequency or peak amplitude of these disturbances can only be measured. Certain characteristics are static features and specific voice signal attributes across time. Dynamic qualities (short-term assessments) are far more informative in terms of sound associates of perceptual components of speech quality that are critical for sickness diagnosis [22]. Dynamic properties show fluctuations in the temporal structure of the excitation signal, whereas fixed characteristics do not. Short-term mel occurrence cepstral coefficients (MFCC) are often used in nonparametric approaches centered on the magnitude spectrum of dialogue [23–25]. The attributes indicated above can be engaged safely for a substantial-scale, quick evaluation of usual and bizarre vocals [26]. Following that, the feature vectors are loaded into a new categorization prototype [27, 28] using multitaper MFCC characteristics and a Gaussian mixture model- (GMM-) based classifier for recognizing chaotic audio signals. [29] built an SVM (support vector machine) for identifying binary pathological conditions using characteristics gathered by inspecting diverse regularity bands with correlation tasks. [30] utilizes ANN (artificial neural network) and SVM (support vector machine) techniques for categorization.

Most studies [31, 32] focus on using audio of consistent vowel /a/ captured in an experimental setting for their research, whereas others [33, 34] focus on the combination of vowels. [32] establishes a high value using 200 continuous vowel /a/ recordings. Other studies [29, 30, 35] use the mixture of vowels /a/, /i/, and /u/ to obtain high precision while disregarding pathological causes. [29] develops a database with three categories of speech pathology models in a binary classification paradigm. While such a clinically insightful data gathering approach may not be a viable choice to utilize in a home-like situation for the nonappearance of a health professional, these methods create a reduced binary classification job to detect only one disease-specific speech problem design. As a result, the scientific community usually overlooks numerous unusual illnesses. This project, on the other hand, employs a big-scale Saarbruecken Voice Database (SVD) [11] that includes both clarifications of vowels similar to /a/ and normal daily interactions by speakers from 71 diverse disease-specific pathology circumstances, presenting a comparatively new and extra difficult task of multiclass categorization.

Deep learning-based vocal pathology detection algorithms recently reached great accuracy [34, 36, 37]. Deep learning models were suggested or imported from image processing programs [8]. In general, such systems transform time-domain sound inputs into spectrograms that may be seen as pictures. VGG-16, AlexNet [38], and CaffeNet were among the frameworks employed in speech pathology studies [39].

## 3. Materials and Methods

As can be seen, Figure 1 depicts the model's whole training pipeline. We started with data collection. The speech pathology database is chosen and given for feature extraction. It extracts vital features for training the model to discriminate pathological sounds from healthy. Frequency domain features are more discriminative than time-domain features and provide deeper insight into the signal-articulation relationship. This study focused on chroma, mel spectrograms, and mel frequency cepstral coefficient (MFCC) features. These feature sets were used to train and test the model.

Figure 2 shows a detailed series of experiments. The complete dataset was split into two collections: a dataset comprising solely “/a/” on the medium pitch and a dataset of voice samples of all the “/a/”, “/i/”, and “/u/” on low, medium, and high pitches. In experiment 1, we built models for these two datasets to categorise audio signals as diseased or healthy. Further experiments were carried out only on different pitches of “/a/”, “/i/” and “/u/” voice samples. Experiment 2 created different (pathological/healthy) models for male and female voices. As part of the second series of studies, we isolated some pathologies from the dataset, built separate (pathological/healthy) models for them, and assessed their performance. Finally, we created a multiclass classification model for two diseases from the dataset. The models follow the same development procedure: feature extraction, feature vector creation, DNN training, and model evaluation.

### 3.1. Dataset

We used the Saarbruecken Voice Database (SVD) for this study [40]. This database contains an extensive collection of normal and pathological speech samples from over 2000 people, all taken in the same context. The dataset includes average, high, and low pitch pronunciations of the vowels /i/, /a/, and /u/, as well as the German sentence “Guten Morgen wie geht es Ihnen?”. The voice samples are 1 to 3 seconds long and captured at 50 kHz with 16-bit resolution. The entire dataset comprises records of 8878 healthy individuals (3360 men and 5518 women) and 17,589 individuals (8149 men and 9440 women) with more than 50 pathologies (Figure 3). 10% of the data is allotted for testing.

Figure 4 shows a visualization of some of the sample audio files. An audio file can be represented as a time series, with the amplitude of the audio waveform as the dependent axis. All information needed to construct features for our model comes from the waveform of the audio signal. The shape of a waveform, on the other hand, does not carry enough discriminating information; therefore, we must change it into a more usable form.  Figure 5 shows the spectrogram of the sample images in the dataset. The graph has two geometric dimensions: one axis represents time, while the other axis indicates frequency; the intensity or color of each point in the graphic provides a third dimension representing the amplitude of a given frequency at a certain time (on a decibel scale).

### 3.2. Feature Extraction

The initial stage in any automatic speech recognition system is to extract features or identify the audio signal components that are useful for detecting linguistic content while ignoring everything else, such as background noise and emotion. Major audio features that help distinguish different audio classes are as follows.

- Chroma features/chromagram
- Mel spectrogram
- Mel frequency cepstral coefficient (MFCC)

#### 3.2.1. Chroma Features/Chromagram

Pitch is a feature of any sound or signal that allows the frequency-related scale to order files. There are 12 different pitch classes in an audio recording. These pitch class profiles are used to analyse audio files. The word “chroma feature” or “chromagram,” also known as “pitch class profiles,” refers to the twelve various pitch classes [41]. At each time frame, the chroma representation shows the intensity of each of the 12 various musical chromas of the octave. Each dimension of a twelve-element vector describing the intensity associated with a given semitone makes up the chroma characteristics regardless of the octave. The chroma feature vector is a 12-element vector that depicts how much energy each of the 12 pitch classes contributes to the whole audio signal. Waveform chromagrams, constant-Q chromagrams, and chroma energy normalized statistics (CENS) chromagrams are the three most common types of chromagrams. The current study focuses on the waveform chromagram generated from the audio signal's power spectrogram.

Figure 6 shows different types of chromagram in which we have used different scales to classify the pitch classes under the audio file. The different colors correspond to different pitch classes.

#### 3.2.2. Mel Spectrogram

A spectrogram depicts the amplitude or loudness of the audio stream overtime at various frequencies in a waveform. It is formed by breaking down the sound duration into smaller time segments and detecting the frequencies present in each segment by creating the Fourier transform of each. Finally, these Fourier transforms were combined to form a spectrogram. The plot shows frequency (*y*-axis) vs. time (*x*-axis), with the amplitude of each frequency shown by a heat map. The higher the signal's energy, the brighter the color, as the concentration of sound around those specific frequencies. The dark color in the plot indicates an empty/dead sound. Thus, a spectrogram helps to understand the shape and structure of audio even without listening to it. However, the spectrograms fail to show the amplitude differences at higher frequencies. This occurs in human audio perception as well. Most of what humans can hear is limited to a small range of frequencies and amplitudes. Our hearing is not linear; it operates on a linear scale.

An ideal audio feature should include time-frequency representation and perceptually relevant amplitude and frequency representation. Unfortunately, the perceptually relevant frequency representation is missing from the spectrogram. However, this can be accomplished using mel spectrograms and the mel scale. A logarithmic transformation of a signal's frequency is the mean scale. The mel spectrogram [42] was created to display audio information closely to how humans perceive it. The underlying notion behind this transformation is that humans perceive that sounds of equal distance on the mel scale are of the same length. Therefore, lower frequencies (Hz) have a larger space between them in mels, whereas higher frequencies (Hz) have a smaller distance between them, strengthening their human-like qualities. Mel spectrograms visualize audio signals on the mel scale instead of the frequency domain as in spectrograms. The equation for converting the frequency in Hz to frequency in Mel [43] is shown.

(1) $$\begin{array}{c} m=2595\;\log_{10}\left(1+\frac{f}{700}\right), \end{array}$$

where *f* denotes the physical frequency in Hz and *m* denotes the perceived frequency in mel scale.

The corresponding inverse operation [43] is given:

(2) $$\begin{array}{c} f=700\left(10\frac{m}{2595}-1\right), \end{array}$$

where *m* denotes the frequency in mel scale and *f*  denotes the frequency in Hertz (Hz).

The critical differences between the mel spectrogram and the standard spectrogram are as follows:

1. The mel scale replaces the frequency on the *y*-axis
2. Instead of amplitude, decibels are used to indicate the colors

After passing through numerous mel filter banks, the original audio waveform was turned into a mel spectrogram. Each audio is given a 128-length feature vector by 128 mel filter banks.  Figure 7 shows a mel frequency representation for healthy and pathological male and female voices.

#### 3.2.3. Mel Frequency Cepstral Coefficients (MFCCs)

The sound produced is determined by the form of the vocal tract. It manifests itself in the short-time power spectrum's envelope, and MFCCs' task is to reflect this envelope appropriately. They were introduced by Davis and Mermelstein [23] in the 1980s and were state of the art until then.

The MFCC formation is shown in Figure 8. Several small frames are created from the original audio input. First, calculate the power spectrum's periodogram estimate for each frame, then apply the mel filter bank to the power spectra, and add the energy in each filter. The logarithmic function is applied to all filter bank energies, followed by a discrete cosine transform to create MFCCs. The detailed explanation of the procedure is given below.

First, convert the audio signal into several frames. *s*(*n*) is our time-domain signal and is converted to *s*_*i*_(*n*) when it is framed, where *i*  indicates the number of the frame. The discrete Fourier transform of the frame is shown [44].

(3) $$\begin{array}{c} S_{i}\left(k\right)=\overset{N}{\underset{n=1}{\sum }}s_{i}\left(n\right)h\left(n\right)e^{-j2\pi kn/N\;}\;1\leq k\leq K, \end{array}$$

where *S*_*i*_(*k*) is the DFT of the frame, *h*(*n*) is a hamming window of *N*  sample length, and *K* is the length of DFT. The periodogram estimate of the power spectrum for the *s*_*i*_(*n*) is given in

(4) $$\begin{array}{c} P_{i}\left(k\right)=\frac{1}{N}{\left|S_{i}\left(k\right)\right|}^{2}, \end{array}$$

where *P*_*i*_(*k*)  is the periodogram estimate of the power spectrum and *N* is the sample length of the hamming window.

Then, compute the mel scale filter bank. To produce MFC, we transformed the logarithmic mel spectrogram back to the time domain. The cepstral representation offers the signal's local spectral properties for frame analysis. Because the mel spectrum coefficients are real numbers, we translate them to the time domain using the discrete cosine transform (DCT), which removes the pitch contribution [45]. MFCC features are the coefficients that make up the mel frequency cepstrum as a whole. The MFCCs are frequently employed in automatic speech and speaker recognition because they carry crucial information about the signal structure [46, 47].  Figure 9 presents a visual representation of MFCC features of healthy and pathological male and female voices.

### 3.3. Deep Neural Network (DNN) Architecture

The designed neural network (Figure 10) comprises five layers (1 input, 1 output, and 3 hidden). The extracted feature vector was 180 dimensions (12 chroma, 128 mel spectrogram, and 40 MFCC). The complete feature vector was normalized before being fed into the neural network design. The label vector was binary because our goal was to classify the audio stream into healthy and diseased categories (healthy vs. unhealthy). The first hidden layer is designed to accept the 180-dimensional feature vector with 100 processing elements (PE). The nonlinear ReLU function was activated, followed by a dropout layer. Dropout [48] is a technique for preventing overfitting in deep neural networks. By randomly removing nodes from the network during training, the network nodes will not coadapt with surrounding nodes, resulting in greater network generalization. We specified a hyperparameter dropout rate when creating the dropout layer, which describes how many nodes to keep at each layer. The dropout only applies to training when we set Training = True since we need all node contributions during inference. The second and third hidden levels followed the same pattern of design. The output layer consists of a single node, and the activation function is also Sigmoid as it performs best on binary classification. The detailed architecture is as shown in Figure 11

### 3.4. Training Setup

By employing the Librosa [49] library and a sampling rate of 50000 Hertz, each audio waveform is processed to yield chroma, mel spectrogram, and MFCC characteristics. It generated feature values for all short-time Fourier transform (STFT) frames, and we created a feature array by taking the mean of each column of the resulting matrix. The scikit-learn [50] library's StandardScaler() function is used to scale the feature vector to make the standard deviation of values equal to 1.

TensorFlow Keras [51] framework is used to construct the architecture, using the sequential function written in Python. The layers were created using the TensorFlow Keras layer library's Dense Dropout Activation functions. The total number of trainable parameters in this DNN was 59,801. We employed the Adam algorithm [52] for gradient-based optimization and the binary cross-entropy loss function used during our proposed model training. With a batch size of 32, the network is meant to run for 100 epochs. Validation accuracy was retained as a checkpoint, and the weights of the best epoch were saved. A 32 GB NVIDIA Quadro P1000 GPU was used for the training.

## 4. Results

Even though the entire collected dataset contains recordings of vowels /a/, /i/, and /u/ in normal, high, and low pitches, as well as an appropriate sentence, we chose to analyse the patient's voice quality using only vowels because they avoid linguistic artifacts and are commonly used in voice assessment applications [53]. Therefore, we trained the DNN model for the entire pathological and healthy database of vowels /a/, /i/, and /u/ in normal, high, and low pitches as a first experiment. Most previous research on diseased voice datasets concentrated on normal pitched vowel /a/ audio recordings [54]. Thus, we made a model with just the vowel /a/ with a standard voice pitch and compared its performance on the test dataset to the previous model (Table 1).

Figure 12 represents the detailed accuracy and error evaluation with the lines drawn for the training and validation phase for the above two models. It is evident that overfitting occurs for the model with only “/a/” vowel.  Figure 13 shows the confusion matrix for the model developed for the entire vowel dataset.

Despite the scholarly interest in the subject, there are still only a handful of continuous speech databases with medical diagnostic annotations that may be used for research. Additionally, there is a minimal scientific study on voice diagnosis utilizing continuous speech [55]. In this sense, we performed our model's prediction on a continuous speech dataset, the German sentence “Guten Morgen wie geht es Ihnen?” from the SVD database, and examined the results in Table 2.

Because the dataset includes information on both male and female genders, the model may become confused due to the extra information. Therefore, we tried to create the model individually for the male and female datasets and compare the results with the model without gender information. The performance analysis of male and female models may be found in Table 3. To better understand the generalization of the model to the unknown data, Table 4 examines the performance of the sentence dataset.

Moreover, we experimented upon the dataset only in relation to the pathological basis. We used a total of 101 dysphonia patients (48 males and 53 females), 140 with chronic laryngitis (57 females and 83 males), 56 dysody (39 females and 17 males), 112 functional dysphonia (76 females and 36 males), 59 vocal cord cordectomy (3 females and 56 males), 68 leukoplakia (41 females and 27 males), and 632 for healthy subjects. The performance analysis for binary classification between selected pathologies on the test dataset is shown in Table 5.

The performance of the model developed for classifying the 3 classes (healthy and pathological, cordectomy, and laryngitis) is shown in Table 6.

## 5. Discussion

The uneasiness of nonautomated methods of vocal pathology testing necessitates using an automated computerised method, which is both convenient for clinicians and favourable to patients [56]. Several studies and developments of machine learning and deep learning algorithms have been conducted to detect vocal disorders. Even though this system's performance is not flawless, they can be used to supplement other laryngoscopy examinations [24]. Inspired by this, rather than focusing on high-accuracy model building with a limited number of pathologies or only a voice with a vowel /a/ in normal pitch, we widen our research towards a more diverse dataset that includes additional pathologies, voice, and pitches. We never examined different features that can successfully discriminate between normal and diseased voices, as [54] did. We only employed the most extensively used feature extractors to train the classifier.

We chose the SVD database because [56] pointed out a drawback of the MEEI database: the healthy and pathological data obtained from various environments. Along with accuracy, we need to understand whether the model learns to distinguish relevant features or overfits on noise or remembers the samples [54], which necessitates data obtained in a consistent setting.

[32] demonstrated that combining classifiers trained on several vowels and pitches resulted in a significant improvement over using simply single vowels since each sound provides the system with unique information. We demonstrated in Table 1 that the model trained on the vowels /a/, /i/, and /u/ pronounced with normal, low, high, and low-high-low intonations outperformed the model trained exclusively on the/a/ vowel with a normal pitch. Moreover, Table 7 demonstrates how our Model beats the previously developed models in the domain with all vowels and only on the vowel /a/. Furthermore, as [57] pointed out, vocal disorders are more difficult to classify from continuous speech than with sustained vowels. On the other hand, our previously trained model shows significant accuracy on continuous speech data extracted from SVD, and it well generalizes to anonymous data and is suitable for applications with constant sentences and vowels (Table 2).

We tried to figure out what elements influence the model's ability to recognize vocal pathology. The underlying factor could be fundamental differences in male and female voice behaviour [33]. The shape of human vocal tracts differs significantly between genders [60], which could lead to various variation features. The preparation and testing information will become increasingly reliable when gender information is included. The performance of the models trained on the female and male voice dataset exceeds vowel prediction and vowel prediction and continuous speech data, as shown in Tables 3 and 4. As a result, it has cleared that gender impacts pathological vs. healthy voice prediction.

To better understand how the suggested model works on various diseases, we selected a few that had a substantial number of examples. Individual diseases exhibit more promising results, as seen in Table 5. [57] suggested that having a model trained in multiple disease classes would be interesting. As a result, we compared our findings with those of [57], on two disorders, dysphonia and laryngitis (Table 8).

Table 5 shows the results of a performance analysis of individual pathologies. Selected pathologies had an accuracy of better than 90%. We built a multiclass classification model using only two pathologies with the highest accuracy, resulting in an accuracy of 86.40% (Table 6). Unfortunately, the SVD dataset has a flaw: the identical voice files were included under multiple pathologies (e.g., dysody, dysphonia, and functional dysphonia). Therefore, we will need a more comprehensive and accurate dataset to classify more disorders. Most previous studies only selected voices with standard speech features, which are straightforward to forecast and clinically interpretable. However, we chose the whole SVD dataset for our research, and it contains sophisticated and difficult voice pattern analysis elements [31]. This was also depicted in Figures 4, 5, 6, 7, and 9), where determining which factors distinguish healthy and diseased voices was extremely challenging. The model's performance on the full dataset is not promising due to the lack of significantly different features for healthy and diseased speech (Table 1). The success of binary classification on selected diseased voices (Table 5) demonstrates that only some pathological voices are considerably different from healthy voices. As a result, including accurate data for both diseased and healthy voices is the only way to increase accuracy. Despite these flaws, the model's generalization to an unknown continuous speech dataset proved surprisingly encouraging.

## 6. Conclusions

Machine learning techniques can be a great way to quickly and easily examine novel signal processing methods that can be used as a health monitoring solution. These approaches were used in several works in vocal pathology detection, but most of them focused on a subset of vowels or pathologies for this job, aimed at achieving high accuracy. Nevertheless, the major drawback is that they fail in generalization to a real-world scenario involving variable voice patterns. The current work developed a customized deep neural network (DNN) algorithm for classifying pathology voices from healthy based on samples from the publicly available Saarbruecken Voice Database (SVD). We also analysed the performance of several models generated with varied datasets acquired through SVD. The results show that the model generated for all vowels /a/, /i/, and /u/ produced at high, low, and normal pitches beat the model developed exclusively for /a/ vowel of a normal pitch. Incorporating gender data can also improve the model's accuracy by 88%. The model developed with data for specific disorders was also 96.77% accurate (cordectomy vs. healthy voice). Additionally, the generated model had a 70.32% accuracy on an entirely unknown German sentence dataset, “Guten Morgen wie geht es Ihnen?”, extracted from SVD and kept separately. The result gave us confidence that, despite the model's lower accuracy, the model may be used in real-time clinical applications where variable pathologies, voices, and pitch are involved.

Thus, our future work will incorporate more accurate data from other publicly available datasets and update more accurate data from other publicly available datasets and update the model to learn meaningful features to produce more accurate results.

## Figures and Tables

**Figure 1:** The block diagram for the pathological voice classification.

**Figure 2:** The block diagram for the pathological voice classification.

**Figure 3:** Distribution of male and female voices in the dataset.

**Figure 4:** Waveforms of healthy and pathological male and female voices.

**Figure 5:** Spectrogram of male and female healthy and pathological voices.

**Figure 6:** Chromagrams of healthy and pathological male and female voices.

**Figure 7:** Mel spectrograms of healthy and pathological male and female voices.

**Figure 8:** The overall process of MFCC.

**Figure 9:** MFC coefficients of healthy and pathological male and female voices.

**Figure 10:** Model architecture.

**Figure 11:** Detailed model architecture.

**Figure 12:** Accuracy and error evaluation of DNN models in training and validation phase: (a) DNN model on /a/, /i/, and /u/ on low, high, and medium pitch and (b) DNN model on /a/ on medium pitch.

**Figure 13:** Confusion matrix of DNN model for the entire vowel dataset.

**Table 1:** The performance comparison of models with the entire vowel voices in the dataset and only the vowel /a/.

Model	Accuracy	F1 score	Recall	Precision
/a/, /i/, and /u/ on low, high, and medium pitch	77.49%	82.21%	83.78%	80.70%
Only /a/ on normal pitch	73.83%	70.47%	69.94%	71.40%

**Table 2:** Performance on the continuous speech dataset.

Model	Accuracy	F1 score	Recall	Precision
/a/, /i/, and /u/ on low, high, and medium pitch	70.32%	78.37%	78.95%	77.80%

**Table 3:** Performance of the pathology detection model trained with gender information on test data.

Model	Accuracy	F1 score	Recall	Precision
Female, i, o, and u pitch	80.63%	77.48%	76.25%	80.02%
Male, i, o, and u pitch	88.01%	80.72%	79.20%	82.63%

**Table 4:** Performance of the pathology detection model trained with gender information on continuous sentence dataset.

Model	Accuracy	F1 score	Recall	Precision
Female voice: /a/, /i/, and /u/ on low, high, and medium pitch	95.66%	96.73%	97.79%	95.68%
Male voice: /a/, /i/, and /u/ on low, high, and medium pitch	72.38%	82.37%	90.44%	75.63%

**Table 5:** Performance of the designed DNN with different pathologies.

Pathology	Accuracy	F1 score	Recall	Precision
Dysphonia × healthy	85.71%	68.12%	64.50%	83.07%
Cordectomy × healthy	96.77%	94.47%	91.66%	98.07%
Dysody × healthy	81.25%	78.18%	76.92%	88%
Functional dysphonia × healthy	86.04%	85.97%	85.97%	85.97%
Laryngitis × healthy	93.87%	93.48%	93.07%	93.99%
Leukoplakia × healthy	89.06%	70.03%	65%	94.26%

**Table 6:** Performance of the designed DNN for the multiclass problem with test data.

	Accuracy	F1 score	Recall	Precision
Healthy, cordectomy, and laryngitis	86.40%	82.95%	80.93%	85.52%

**Table 7:** Performance comparison of the model trained on all vowels and all pitches with previous works.

Model	Accuracy
Ours	77.49%
[58]	77.21% (all vowels)
[59]	73.3% (only /a/)
[54]	68.08% (only /a/)

**Table 8:** Comparison of performance for continuous speech prediction.

	Models	Precision	F1 score
Dysphonia × healthy	Ours	83.92%	82.10%
	[57]	63%	63%
Laryngitis × healthy	Ours	80.57%	78.77%
	[57]	67%	67%

## Data Availability

The dataset used in this study is available at http://www.stimmdatenbank.coli.uni-saarland.de/help_en.php4.
